# Effects of Propofol Intravenous Anesthesia on Serum NGF, S100B Protein, and Immune Function in Patients with Bladder Cancer after Resection

**DOI:** 10.1155/2022/5409323

**Published:** 2022-08-28

**Authors:** Xiaohong Guan, Qingxiong Peng, Yongping Liu, Jiansong Wang

**Affiliations:** ^1^Department of Anesthesiology, The First Hospital of Changsha, Changsha, 410011 Hunan, China; ^2^Department of Anesthesiology, Hunan Provincial People's Hospital, The First Affiliated Hospital of Hunan Normal University, Changsha, 410005 Hunan, China; ^3^Department of Urology, Hunan Provincial People's Hospital, The First Affiliated Hospital of Hunan Normal University, Changsha, 410005 Hunan, China

## Abstract

**Objective:**

To explore the efficacy of intravenous propofol anesthesia on patients with bladder cancer after resection, as well as its effect on cognitive and immune function.

**Methods:**

Patients with bladder cancer and received resection of bladder cancer at our hospital from May 1, 2019, to November 30, 2021, were retrospectively retrieved and included in this study. The included patients were summarized into group A (isoflurane) and group B (intravenous propofol). The anesthesia intervention effect, serum NGF level, serum S100B protein level, and immune function before surgery, 6 h after surgery, 1 d after surgery, and 3 d after surgery were compared between the two groups.

**Results:**

Eighty-six patients were retrieved. The anesthesia intervention effective rate of patients in group B was significantly higher than that of patients in group A (*P* < 0.01). The serum NGF and S100B of patients in both groups were significantly lower on postsurgical day 1, but in the trend to returning to those before intervention level on day 3. There were also fluctuations in immune function represented by changes in CD3+, CD4+, CD8+, and CD4+/CD8+ T cells, which showed return of function by postsurgical day 3.

**Conclusion:**

The anesthetic effect of intravenous propofol in patients with bladder cancer resection is significantly more satisfactory than isoflurane, with a transient effect on serum NGF and S100B protein levels and patients' immune function, which suggests that intravenous propofol can be widely used for general anesthesia in clinical practice.

## 1. Introduction

Propofol and other intravenous (IV) sedative-hypnotic medications are commonly used for general anesthesia. Some studies have shown that anesthesia medications can cause postoperative cognitive dysfunction and immune dysfunction in old patients, which will seriously affect the quality of life of patients after surgery [1]. Patients with bladder cancer are diagnosed at an average of 73 years old, which is a typical group of aged population [2]. The influence of different anesthesia regimens on the cognitive function and immune function of patients with bladder cancer resection is still concerned by clinicians around the world [3].

Some studies have shown that both serum NGF and S100B protein are key markers for evaluating whether patients' postoperative cognitive function is impaired or not [4, 5]. It was found that propofol has a rapid onset of anesthesia effect, few adverse effects, and also a minor impact on the cognitive function of patients [6, 7]. Therefore, we analyzed the anesthesia effect of propofol, its impact on serum NGF, S100B protein levels, and immune functions in patients who received bladder cancer surgery.

## 2. Materials and Methods

Patients with bladder cancer undergoing resection of bladder cancer who were treated at our hospital from May 1, 2019, to November 30, 2021, were included in this study. Patients in group A received isoflurane during the resection, while patients in group B received intravenous anesthesia with propofol. This study was approved by the institutional ethical committee of our hospital. All the included patients and their families were informed about the study and actively signed the consent form.

Inclusion criteria are as follows: (1) all the included patients met the corresponding criteria for bladder cancer resection [8], (2) aged between 18 and 85 years, and (3) the clinical data of all included patients were complete.

Exclusion criteria were as follows [9]: (1) patients had a history of allergy to the anesthetic drugs in this treatment plan, (2) patients had severe organ dysfunction, and (3) patients had severe respiratory diseases.

First, the patient was given an intramuscular infusion of atropine (Tianjin Jinyao Pharmaceutical Co., Ltd., H12020384) 0.5 mg before surgery. Secondly, the clinical signs of the patient were monitored immediately after entering the operating room, and 0.04 mg/kg midazolam (Yichang Renfu Pharmaceutical Co., Ltd., approved by H20065729) and 0.4 μg/kg fentanyl (Jiangsu Enhua Pharmaceutical Group Co., Ltd., National Medicine Zhunzi H19990027) were given for anesthesia induction, and then, tracheal intubation was performed to assist ventilation. Then, patients in group A were given 1%-3% isoflurane (Shanghai Hengrui Pharmaceutical Co., Ltd., approved by H20070172) by inhalation to maintain anesthesia, while patients in group B were given 4 mg/kg/h propofol (Xi'an Libang Pharmaceutical Co., Ltd., Chinese Medicine Zhunzi H19990282) intravenous infusion to maintain anesthesia. Finally, vecuronium bromide (Hubei Keyi Pharmaceutical Co., Ltd., H20084581) and fentanyl were intermittently administered to maintain anesthesia during the operation, and the infusion was terminated 30 minutes before the completion of the operation. Before and after the intervention, 5 ml of venous whole blood was collected from all of the included patients in the fasting state in the morning for various experiments, which was aliquoted and either used freshly or placed in a -80°C refrigerator for later use.

### 2.1. Evaluation of the Effect of Anesthesia Intervention

Remarkable effect: the patient's anesthesia induction state was stable, the depth of anesthesia maintenance was reasonable, and the state was stable during recovery. Normal effect: the patient's anesthesia induction state was relatively stable, the depth of anesthesia maintenance was reasonable, and mild agitation occurred during recovery. Poor effect: the patient's state of anesthesia induction was unstable, the depth of anesthesia maintenance was unreasonable, and severe agitation occurred during recovery. The total intervention effective rate = (significant + general)/total number of cases × 100% [10, 11]. The American Society of Anesthesiologists (ASA) physical status classification system was used to evaluate the physical status of enrolled patients [12].

### 2.2. Detection of Serum NGF Levels

The serum nerve growth factor (NGF) levels of all included patients were detected before surgery, 6 h, 1 d, and 3 d after surgery by enzyme-linked immunosorbent assay (ELISA). The kit was purchased from Shanghai Kanu Biotechnology Co., Ltd. and operated in strict accordance with the instructions to control the intrabatch variation < 10% and the interbatch variation < 15% [13].

### 2.3. Detection of Serum S100B Protein Level

The serum S100B protein levels of all included patients were checked before the operation, 6 h, 1 d, and 3 d after operation by (ELISA). The kit was purchased from Shanghai Kanu Biotechnology Co., Ltd. and operated in strict accordance with the instructions to control intrabatch variation < 10% and interbatch variation < 15% [14].

### 2.4. Assessment of Immune Function

Each patient's whole blood sample (2 ml) was treated with heparin and put into sterile EP tubes, and one volume of PBS was added to dilute the blood. The total live cell concentration was adjusted to 2 × 10^6^ in DMEM medium (Youkang Hengye Biotechnology (Beijing) Co., Ltd., China), followed by addition of anti-CD3+, CD4+, and CD8+ antibodies (1 μg per 10^6^ cells, Abcam, China) at room temperature in the dark for 20 min. The samples were then washed three times with PBS buffer and analyzed by flow cytometry (Navios, Beckman Coulter, USA).

### 2.5. Statistical Methods

The data in this study were analyzed by SPSS21.0 software package (IBM Corp., Armonk, N.Y., USA). The enumeration data (%) were analyzed by *χ*^2^ test, and the measurement data (mean ± SD) were analyzed by *t* test. A *P* < 0.05 (2-sided) means the difference is significantly different.

## 3. Results

### 3.1. Comparison of the Effect of Anesthesia Intervention

A total of 86 qualified patients (43 cases in group B and 43 matched cases in group A) were retrieved. The average age of patients was 57.87 ± 5.43 years in group A and 58.23 ± 5.33 years in group B. There was no difference in gender, age, BMI, or ASA rating between the two groups (*P* > 0.05 for all comparisons). The general data of the patients included in this study are shown in Table 1.

The total intervention effective rate of patients in group B was significantly higher than that of patients in group A (88.37% vs. 74.41%, *P* < 0.01, Table 2).

### 3.2. Comparison of Serum NGF Levels

Before surgery, the serum NGF level of patients in group B (348.21 ± 36.83) was not significantly different from that of patients in group A (332.38 ± 34.67) (*t* = 1.664, *P* > 0.05); 6 h and 1 d after surgery, the serum NGF levels of patients in group B were significantly lower than those of group A patients (271.21 ± 37.83 and 287.78 ± 30.34 vs. 282.38 ± 41.67 and 295.12 ± 37.56, *t* = 3.764, 2.275, *P* < 0.01, respectively). But 3 days after surgery, the serum NGF level of group B patients was not significantly different from that of group A patients (336.41 ± 33.26 vs. 328.34 ± 36.41, *t* = 1.363, *P* > 0.05) and has returned to the preoperative level (Table 3).

### 3.3. Comparison of Serum S100B Protein Levels

Before surgery, the serum S100B protein level of patients in group B was not significantly different from that in patients in group A (0.37 ± 0.33 vs. 0.38 ± 0.32, *t* = 0.223, *P* > 0.05); 6 h and 1 d after surgery, the serum S100B protein levels of patients in group B were significantly higher than those of patients in group A (0.81 ± 0.53 and 0.68 ± 0.44 vs. 0.74 ± 0.47 and 0.42 ± 0.32, *t* = 0.564, 0.575, *P* < 0.01, respectively). But 3 days after surgery, the serum S100B protein level of patients in group B was not significantly different from that in patients in group A (0.36 ± 0.34 vs. 0.37 ± 0.33, *t* = 0.225, *P* > 0.05) and has returned to the preoperative level (Table 4).

### 3.4. Comparison of Immune Function

Before intervention, the CD3+, CD4+, CD8+, and CD4+/CD8+ cells of group B patients were similar as those of group A patients (61.05 ± 7.36 vs. 61.01 ± 8.23, 37.07 ± 4.24 vs. 37.64 ± 4.18, 25.05 ± 2.68 vs. 24.07 ± 3.05, and 1.66 ± 0.13 vs. 1.63 ± 0.14, *P* > 0.05, respectively), whereas after intervention, the CD3+, CD4+, CD8+, and CD4+/CD8+ of patients in both groups were significantly lower on day 1, but in the trend to returning to those before intervention level on day 3 (Table 5).

## 4. Discussion

Cognitive impairment after resection of bladder cancer is commonly seen, especially in older patients, and the incidence is usually between 6% and 62% [15, 16]. Some researchers have claimed that cognitive function has a certain relationship with the central cholinergic system in patients, and serum NGF and S100B proteins are both serum factors that are closely related to cognitive dysfunction in patients [17, 18]. Our study indicates that propofol is effective for anesthesia intervention, which also has only transient on the serum NGF and S100B protein levels. The reason may be that propofol does not disturb the production of inflammatory chemokines in the body, thereby improving the function of the central cholinergic system [19].

CD4^+^ and CD8^+^ T cells, as key components of the immune system, can effectively reflect the changes in immune function in the body [20–22]. In this study, we found that after propofol application in groups A and B, all CD3+, CD4+, CD8+, and CD4+/CD8+ T cells changed significantly on day 1 compared with those before propofol application, then in the trend of recovery on day 3, which indicated that intravenous anesthesia by propofol had only transient effect on the immune function of patients and this was helpful for the recovery of postoperative immune function of patients. The reason for this may be that propofol is less irritating to the patient's body and will not cause too much stress and inflammatory response to the patient [23, 24].

Although propofol is an effective anesthetic reagent and has little effect on cognitive and immune functions, it still needs to be evaluated in severe clinical conditions, such as fulminant hepatitis, hypoxia brain injury, preterm labor, or intrauterine infections during pregnancy [25–33].

All in all, the anesthesia intervention effect of propofol intravenous anesthesia in patients undergoing bladder cancer resection is remarkable, with little effect on serum NGF and S100B protein levels, and does not interfere with the recovery of patients' immune function, suggesting that it can be widely used in clinical practice.

## Figures and Tables

**Table 1:** Comparison of clinical characteristics of the two groups of patients.

Group	Case	Gender (male/female)	Age (years old)	BMI (kg/m^2^)	ASA rating		
					I	II	III
Group A	43	24/19	57.87 ± 5.43	25.57 ± 4.32	25	12	6
Group B	43	25/18	58.23 ± 5.33	25.74 ± 4.44	26	13	4
*χ* ^2^/*t*		0.157	0.252	0.356	0.327		
*P*		0.787	0.675	0.588	0.554		

**Table 2:** Comparison of the effect of anesthesia intervention between the two groups (*n* (%)).

Group	Remarkable	Normal	Poor	Total intervention effectiveness
Group A (*n* = 43)	19 (44.18)	13 (30.95)	11 (26.19)	32 (74.41)
Group B (*n* = 43)	24 (55.81)	14 (33.33)	5 (11.91)	38 (88.37)
*χ* ^2^	—			7.325
*P*	—			<0.01

**Table 3:** Comparison of serum NGF levels between the two groups of patients after intervention ($\bar{x}\pm s$).

Group	Group A (*n* = 43)	Group B (*n* = 43)	*t*	*P*
Before surgery	332.38 ± 34.67	348.21 ± 36.83	1.664	>0.05
6 h after surgery	282.38 ± 41.67	271.21 ± 37.83	3.764	<0.01
1 d after surgery	295.12 ± 37.56	287.78 ± 30.34	2.275	<0.01
3 days after surgery	328.34 ± 36.41	336.41 ± 33.26	1.363	>0.05

**Table 4:** Comparison of serum S100B protein levels between the two groups of patients after intervention ($\bar{x}\pm s$).

Group	Group A (*n* = 43)	Group B (*n* = 43)	*t*	*P*
Before surgery	0.38 ± 0.32	0.37 ± 0.33	0.223	>0.05
6 h after surgery	0.74 ± 0.47	0.81 ± 0.53	0.564	<0.01
1 d after surgery	0.42 ± 0.32	0.68 ± 0.44	0.575	<0.01
3 days after surgery	0.37 ± 0.33	0.36 ± 0.34	0.225	>0.05

**Table 5:** Comparison of the immune function of the included patients between the two groups ($\bar{x}\pm s$).

Group	Group A (*n* = 43)	Group B (*n* = 43)
CD_3_^+^		
Before intervention	61.05 ± 7.36	61.01 ± 8.23
1 d after intervention	48.06 ± 9.13^^^	50.14 ± 12.52^^^
3 d after intervention	57.06 ± 8.05^^^	59.14 ± 10.38
CD_4_^+^		
Before intervention	37.07 ± 4.24	37.64 ± 4.18
1 d after intervention	27.18 ± 6.33^^^	29.25 ± 7.61^^^
3 d after intervention	34.18 ± 5.19^^^	35.75 ± 5.64
CD_8_^+^		
Before intervention	25.05 ± 2.68	24.07 ± 3.05
1 d after intervention	20.60 ± 3.17^^^	20.41 ± 2.32^^^
3 d after intervention	23.60 ± 3.35^^^	23.41 ± 2.61
CD_4_^+^/CD_8_^+^		
Before intervention	1.66 ± 0.13	1.63 ± 0.14
1 d after intervention	1.38 ± 0.15^^^	1.37 ± 0.25^^^
3 d after intervention	1.48 ± 0.17^^^	1.57 ± 0.16^∗^

Note: compared with the control group, ^∗^*P* < 0.05; compared with before treatment, ^^^*P* < 0.05.

## Data Availability

The data used to support the findings of this study are available from the corresponding author upon request.
